# Improved Calculation Method of TAD for Intertrochanteric Fractures

**DOI:** 10.1155/2022/7729959

**Published:** 2022-12-06

**Authors:** Jialong Wang, Anhua Long, Xuefei Wang, Yakui Zhang, Dacheng Han

**Affiliations:** Department of Orthopedics, Beijing Luhe Hospital, Capital Medical University, Beijing 101149, China

## Abstract

**Purpose:**

To investigate the relative position of femur fixed screws using intramedullary systems for intertrochanteric fractures and to improve the accurate measurement method of the tip-to-apex distance (TAD) while providing a theoretical basis for the clinical treatment of such fractures.

**Methods:**

In the anteroposterior (AP) radiographs of the hip joint, the femoral neck axis through the femoral head geometry point was designated as the *X*-axis, while the line perpendicular to the *X*-axis passing through the femoral head geometry point was designated as the *Y*-axis. In the lateral radiographs of the hip joint, the line perpendicular to the *X*-axis passing through the femoral head geometry point was identified as the *Z*-axis. The head of the nail tip's location projected on the three axes was described as *A*_AP_, *B* in the AP radiographs; and *A*_LAT_, *C* in the lateral radiograph. The TAD was described as *X*_AP_ and *X*_LAT_. The radius of the femoral head was *D*. All distance units were expressed in mm.

**Results:**

When the lateral projection angle was standardized, the *A*_AP_ was equal to the *A*_LAT_, while the *X*_AP_^2^=*B*^2^+(*D* − *A*_AP_)^2^ and *X*_LAT_^2^=*C*^2^+(*D* − *A*_LAT_)^2^. When the lateral projection angle was not standardized, the value of *C* had no significant change; however, the (*D* − *A*_LAT_) value changed.

**Conclusions:**

The measurement value did not match the actual values of TAD when the lateral projection angle was not standardized, possibly leading to a misinterpretation during clinical work. The *X*_LAT_ should be amended using the formula *X*_LAT_^2^=*C*^2^+(*D* − *A*_AP_)^2^.

## 1. Introduction

Intertrochanteric fractures are one of the most common fractures in elderly patients [1]. According to the United States National Statistics, there are 2,50,000 new cases of intertrochanteric fractures annually. Among these, 90% of patients are elderly patients aged above 70 years and 30% are generally hospitalized [1–3]. The most commonly used treatment of intertrochanteric fractures is the intramedullary fixation system, particularly for unstable fractures of AO type 31-A2.2 or above [4, 5].

When intertrochanteric fractures are treated using an intramedullary fixation system, we should fully assess the patient's fracture type, bone quality, compliance, and complications, and also select the appropriate internal fixation according to the patient's specific situation. Moreover, the internal fixation system should be placed at an appropriate location of internal fixation to achieve the ideal therapeutic effect. This requires a complete evaluation and system to ensure the quality of treatment [6, 7]. Among many evaluation methods, the tip-to-apex distance (TAD) is one of the most commonly used evaluation indicators [6–8].

Baumgaertner [8] proposed the concept of TAD in 1995, which is the value obtained by sum of the distance between the AP view and lateral view in radiographic plates, the femoral head vertex and the screw vertex with magnification, TAD=*X*_AP_+*X*_LAT_, <25 mm (Figure 1). This is a calculation method based on two-dimensional space, which has been widely used to evaluate the relative position of the posterior screw during the operation of intertrochanteric fracture and to provide a reference for the treatment quality and prognosis of patients.

TAD is the sum of two projection lines perpendicular to each other, not the true distance between the screw tip and the apex of the femoral head. Therefore, Baumgaertner also used the method of three-dimensional (3D) geometry to calculate the real distance. He found that the real distance is smaller than the sum of the two image distances, the average difference is between 0.49 and 0.82 mm, and the correlation coefficient between them is 0.97. Therefore, it is more convenient to use a simple two-dimensional method to determine TAD values.

However, in clinical work, we found that when the angle of the radiographic lens changed, the relative position of the nail point in the femoral head shown on the radiograph could not accurately reflect the real situation in the patient's hip. When we do the X-ray after surgery, in the anteroposterior (AP) view, the patient should lie on his back on the photographic table, with his lower limbs straightened and his feet tilted inward by 25°. In the lateral view, the patient should lie on the ill side of the photographic table, straighten the lower limb and keep the femur lateral to the table, bend the hip joint on the healthy side at a right angle to the trunk, and the axis of the femoral neck should be perpendicular to the lens direction. I found that as a young person I am, I also had some difficulty trying to stay in this position until the radiation was finished (Figure 2), and even we place a stacked pillow beneath the medial side of the affected thigh, it is also difficult to get a standard lateral view because of body size, pain, etc. Similarly, during surgery, it is difficult to obtain a standard lateral view due to the position of the operative body and the placement of the C-arm. In the process of surgery, many hospitals cannot use software to accurately calculate how to correct the TAD. Therefore, it is difficult for elderly patients with hip fractures to complete a perfect lateral view, both during or after the surgery, that will affect the accuracy of the final TAD.

Thus, we conducted a 3D spatial setting and measurement based on the anatomical structure of the proximal femur to explore the relative position of the head nail during the fixation of intertrochanteric fractures using the intramedullary nail system and improved the accurate measurement method of the TAD to provide a theoretical basis for the clinical treatment of such fractures.

## 2. Materials and Methods

### 2.1. Study Object

We chose the X-ray of the hip joint as the study object. For the AP view, the patient must lie on his back on the photographic table, with his lower limbs straightened and his feet tilted inward by 25°. Moreover, for the lateral view, the patient should lie on the ill side of the photographic table, straighten the lower limb and keep the femur lateral to the table, bend the hip joint on the healthy side at a right angle to the trunk, and the axis of the femoral neck should be perpendicular to the lens direction. We determined the geometric center point of the femoral head using the chordal tangential method (Figure 3).

### 2.2. Construction of the 3D Model

In the AP radiographs of the hip joint, the femoral neck axis through the femoral head geometry point was assigned as the *X*-axis, while the line perpendicular to the *X*-axis passing through the femoral head geometry point was the *Y*-axis. In the lateral radiographs of the hip joint, the line perpendicular to the *X*-axis passing through the femoral head geometry point was demarcated as the *Z*-axis. The head of the nail tip's (tip) location projected on the three axes could be described as *A*_AP_ (*X*-axis), *B* (*Y*-axis) in the AP radiographs, and *A*_LAT_ (*X*-axis), *C* (*Z*-axis) in the lateral radiographs. The TAD was described as *X*_AP_ and *X*_LAT_ in the AP and lateral radiographs, respectively. The radius of the femoral head was *D* (Figure 4). All distance units were expressed in mm. Then, we can calculate the actual value of TAD according to the Pythagorean theorem.

## 3. Results

In the 3D structure, we take the center point as a reference, and the position of the screw tip can be marked by the projection coordinates on the three-axes perpendicular to each other, namely, the *X*, *Y*, and *Z* axes. Therefore, in the tip (*A*, *B*, and *C*), *A* is the distance from the tip to plane *YZ*, *B* is the distance from the tip to plane *XZ*, and *C* is the distance from the tip to plane *XY*. Therefore, *X*_AP_^2^=*B*^2^+(*D* − *A*_AP_)^2^ and *X*_LAT_^2^=*C*^2^+(*D* − *A*_LAT_)^2^.

Under the same magnification rate, as it is easy to take the AP view for the patient, the error between *A*_AP_ values and its actual values is relatively small. But the *X*_AP_, *A*_LAT_, *C*, and *X*_LAT_ will change due to the angle of the radiographic lens. However, in the 3D space, both *A*_AP_ and *A*_LAT_ are the distances from the tip to plane *YZ* and should have equal values. This means *A*_LAT_ = *A*_AP_ in a standard lateral view; therefore, *A*_AP_ can replace *A*_LAT_. However, when we cannot take a standard lateral view, the true distance of the *C* value is smaller than the measurement distance. However, since the value of (*D* − *A*_LAT_)^2^ is much larger than *C*^2^, it has no significant influence on *X*_LAT_; therefore, the measurement value can be used for calculation. However, when the value of (*D* − *A*_LAT_) changes, the change of *X*_LAT_ is relatively large; therefore, *A*_LAT_ should be replaced by *A*_AP_.

## 4. Discussion

The intramedullary nail fixation system is a common choice in the treatment of intertrochanteric fractures. In particular, in unstable intertrochanteric fractures, the intramedullary nail fixation system is preferred for treatment [9, 10]. Currently, common intramedullary nailing systems include a variety of internal fixation systems provided by various manufacturers, such as Gamma III, PFNA, and InterTAN. For stable intertrochanteric fractures, the use of the dynamic hip screws' internal fixation system is currently considered an effective option [11, 12]. The above internal fixation system for the treatment of intertrochanteric femur fractures encounters challenges with the relative position of the head nail in the femoral head during the specific operation and use. If this challenge is not resolved appropriately, it will directly affect the treatment effect and even lead to the serious consequences of internal fixation failure [5, 6]. In clinical practice, the most commonly used indicator to evaluate the relative position of the head nail in the femoral head is the TAD discussed in this study.

Although calTAD has been thought to measure the real TAD data, a study that introduced calTAD appeared in 2012 was identified by Kashigar et al. [13] as the only significant predictor of cutoff. calTAD less than 20.98 mm patients did not see a failure. Contrary to these recent findings, the team's study did not demonstrate the superiority of calTAD over TAD.

TAD and calTAD were proved to be relevant and independent predictors of screw transection probability in peritrochanteric fracture fixation. This does not prove the superiority of calTAD over TAD. From a surgical practice point of view, for young patients with intertrochanteric fractures, we believe that the ideal location for head screws is the central region of the femoral head. In patients with osteoporotic fractures, the ideal location of the head screw is below the center of the femoral head to reduce the risk of osteotomy. Therefore, TAD is still irreplaceable in clinical applications.

Accurate measurement of TAD values intraoperatively and postoperatively is of great value for the outcome of surgery and the prognosis of postoperative patients. Accurate measurements are based on the acquisition of standard AP view and lateral view of the hip, including intraoperative C-arm use and postoperative radiographic imaging of the patient in the correct projection position. In this study, for the AP view, the patient should lie on his back on the photographic table, with his lower limbs straightened and his feet tilted inward by 25°. Moreover, for the lateral view, the patient should lie on the ill side of the photographic table, straighten the lower limb and keep the femur lateral to the table, bend the hip joint on the healthy side at a right angle to the trunk, and the axis of the femoral neck should be perpendicular to the lens direction. Standard AP view is relatively easy to obtain intraoperatively and postoperatively while obtaining standard hip lateral radiographs is challenging due to the lack of accurate reference and the difficulty in positioning and maintaining posture in elderly patients. Therefore, errors are prone to occur in the measurement of TAD or lead to errors in clinical judgment. In this study, we conducted a 3D setting and measurement based on the anatomical structure of the proximal femur to explore the exact position of the head nail in the femoral head during the fixation of intertrochanteric fractures using the intramedullary nail system.

Based on the above understanding, most of the lateral views in clinical work may not be standardized. However, it is highly complicated to measure TAD values through CT using the 3D method. Therefore, to accurately calibrate the relative position of the nail within the femoral head, the geometric center of the femoral head was marked as *A* reference point, and through the geometric center three perpendicular *X*, *Y*, and *Z* axes were demarcated. The reference point was made at any point in the femoral head in these three axes, independent of the projective coordinates (*A*, *B*, and *C*), and indicated to nail tip relative position within the femoral head. Based on this, the measurement of TAD was standardized. According to the Pythagorean theorem, the *X*_AP_ and *X*_LAT_ of TAD can be calculated using Formula (1):

(1) $$\begin{array}{c} X_{AP}^{2}=B^{2}+{\left(D-A_{AP}\right)}^{2},X_{LAT}^{2}=C^{2}+{\left(D-A_{LAT}\right)}^{2}. \end{array}$$

In the calculation of TAD, the magnification of radiographic slices has been well resolved in previous studies [8]. However, there are still some conflicting factors regarding the angle of the radiographic lens. In particular, in the hip, the lateral view is more obvious. In clinical practice, when an internal fixation system is used to treat intertrochanteric fractures, the axis of the head nail and femoral neck generally have an angle, which leads to measurement deviation of *C* and *A*_LAT_ value, which has a great influence on the final calculation results of TAD. In general, the following possibilities may occur. First, when the axis of the head nail is perpendicular to the projection direction, its projection coordinate on the *X*-axis is the largest, and the *A*_LAT_ value is larger than that of the standard lateral view. In the range where the projection direction changes from the standard side to perpendicular to the axis of the head nail, the measured value is larger than that of the standard side. Second, beyond this range, that is, if the projection angle is too skewed, the image will drift and become elongated or shortened, and the TAD cannot be measured normally. In the first case, according to our 3D setting and calculation formula, the *A*_LAT_ becomes larger, and the value of *D* − *A*_LAT_ becomes smaller, resulting in a smaller measurement value of *X*_LAT_ than in the standard case. TAD measurements can be less than 25 mm, and TAD actual values to be more than 25 mm, leading to clinical misjudgment and affecting surgical and patient outcomes. In our study, the *A*_AP_ value was equal to the *A*_LAT_ value when we take the standard AP and lateral views because they all represent the distance from tip to plane of *Y* and *Z* axes. However, the *A*_AP_ value produced less error during the actual radiography; therefore, it could be used as a substitute for the *A*_LAT_ value to correct the *X*_LAT_ value. Then, the calculation formula can be modified as *X*_LAT_^2^=*C*^2^+(*D* − *A*_AP_)^2^. While the true distance of the *C* value is smaller than the measurement distance. However, since the value of (*D* − *A*_LAT_)^2^ is much larger than *C*^2^, it has no significant influence on *X*_LAT_; therefore, the measurement value can be used for calculation.

For example, in this case (Figures 5 and 6), we can measure the values mentioned above from the X-ray of the hip joint. Although in this case, the lateral wall of the proximal femur was not reduced as expected, it did not affect the calculation of TAD. According to the measurement, *X*_AP_ is 14.8 mm, *A*_AP_ is 16.8 mm, *B* is 8.2 mm, *X*_LAT_ is 9.9 mm, *A*_LAT_ is equal to *A*_AP_, *C* is 6.2 mm, and *D* is 29.12 mm. Then, through the classical algorithm, we can get that TAD=*X*_AP_+*X*_LAT_ is finally equal to 24.7 mm, <25 mm. However, according to our improved algorithm, TAD=*X*_AP_+*X*_LAT_= is finally equal to 28.6 mm, >25 mm. This will make a difference in the postoperative X-ray evaluation of patients with intertrochanteric fractures.

Other factors that may influence the measurement of TAD values, such as the location of the projection center and the impact of the rake angle, which were not discussed in depth in this study can be further analyzed in the next study. To sum up, this study set and measured the 3D space based on the anatomical structure of the proximal femur. When the lateral projection angle was not standardized, the measured values of TAD were inconsistent with the actual values of TAD, which might cause clinical judgment errors. *X*_LAT_ should be modified and the calculation formula is *X*_LAT_^2^=*C*^2^+(*D* − *A*_AP_)^2^.

(2) $$\begin{array}{c} TAD=X_{AP}+X_{LAT}=\sqrt{B^{2}+{\left(D-A_{AP}\right)}^{2}}+\sqrt{C^{2}+{\left(D-A_{AP}\right)}^{2}}. \end{array}$$

## Figures and Tables

**Figure 1:** TAD = *X*_AP_ + *X*_LAT_.

**Figure 2:** Position of the patient in radiology after surgery.

**Figure 3:** (a) AP radiographs; (b) lateral radiographs. We have plotted the geometric relations of the three points in different planes.

**Figure 4:** The three-dimensional (3D) structure. We combine the two dimensions obviously into a solid sphere in order to better show the value of TAD.

**Figure 5:** Postoperative X-ray of a patient with intertrochanteric fracture of femur.

**Figure 6:** Calculate the data according to the formula. We can get a more accurate TAD.

## Data Availability

The data used to support the findings of this study are available from the corresponding author upon request.

## Abbreviations

TAD: Tip-to-apex distance
AP: Anteroposterior
3D: Three-dimensional.
